# UPLC/ESI-MS Phytochemical Screening of *Deverra tortuosa* Haematological and Histopathological Studies and Streptozotocin-Induced Diabetes in Rat

**DOI:** 10.1155/2021/4718854

**Published:** 2021-10-28

**Authors:** Fahad A. Alhumaydhi, Abdullah S. M. Aljohani, Eman R. Elsharkawy

**Affiliations:** ^1^Department of Medical Laboratories, College of Applied Medical Sciences, Qassim University, Buraydah, Saudi Arabia; ^2^Department of Veterinary Medicine, College of Agriculture and Veterinary Medicine, Qassim University, Buraydah, Saudi Arabia; ^3^Department of Eco Physiology, Ecology and Range Management Division, Desert Research Center, Mathef El-Mataria 15753, Egypt; ^4^Department of Chemistry, Faculty of Science, Northern Border University, Arar, Saudi Arabia

## Abstract

Herbal plants represent a new source of hypoglycemic antidiabetic drugs; haematological and histopathological studies of methanol extract of *Deverra tortuosa* in streptozotocin-induced diabetic rats were investigated *in vivo*. A single intraperitoneal injection of 160 mg/kg bodyweights of streptozotocin was used to cause diabetes. Blood glucose levels were tested with an AccuCheck Advantage II glucometer and blood glucose test strips. After diabetes was confirmed, animals were orally treated with the extract, metformin, and insulin according to the experimental design. After extract therapy, histological alterations in the pancreas of diabetic rats were investigated. When compared to a control group, daily oral administration of *D. tortuosa* extract (300 mg/kg body weight) plus metformin (100 mg/kg) had a positive effect on blood glucose levels as well as showed an increased number of white blood cells (WBCs) and red blood cells (RBCs). The treatment with the extract for two weeks showed a positive impact on pancreatic histopathological changes in the groups with the diabetic rats. Phenolic fraction of the methanol extract was screened by the liquid chromatography-mass spectroscopy (LC-MS) method, which unveiled the existence of flavonoid compounds and phenolics as kaempferol, rutin, isorhamnetin-3-O-rutinoside, caffeic acid, and 4-hydroxybenzoic acid 4-O-glucoside. The results confirmed the use of the plant as an antidiabetic agent; the research recommended further studies on the plant to use the plant as an antidiabetic drug, where the plant extract also showed improvement in blood parameters.

## 1. Introduction

The use of herbal medicines has increased in the last decade because of their effectiveness, safety, and affordability. WHO recommended the use of traditional plants in the treatment of diabetes. Products isolated from medicinal plants are usually used in the traditional Indian system and have shown clinical antidiabetic activity [1]. One of the dangerous diseases that developed due to irregularities in the metabolism of carbohydrate, protein, and fat is diabetes mellitus which influences insulin hormone. All of this is linked to oxidative stress, which is caused by a rise in free radical levels and a drop in antioxidant defenses [2].

*D. tortuosa* is used as “edible food; its aerial parts are used as fuel wood and have many medical uses. Saudi Arabian plant *D. tortuosa* showed antioxidant, allelopathic, and antifungal activity, used in traditional medicine as a drug for hypertension and against conception [3, 4]. Azzazi et al. described the major compound of essential oil was terpinen-4-ol [5]. *D. tortuosa* is a salt-tolerant plant; it is grown in many phytogeographical habitats in Egypt, in desert wadis, sandy, and stony plains. This plant is dispersed in Egypt, Tunisia, Libya, and Saudi Arabia [6].

*D. tortuosa* (Arabic name is Shabat Elgabal) belongs to Apiaceae family, is an Arabic name, and has an aromatic scent; it is characterized by a high concentration of phytochemical compounds, flavonoids, coumarins, furanocoumarin, glucosides, and terpenes [7, 8]. The plant was pharmacologically active and is used to treat asthma, hepatitis, fever, and diabetes. Ethyl acetate extract of *D. tortuosa* has anti-*Candida* activity and antivirulence activity [9].

The current research was aimed to evaluate the role of plant *D. tortuosa* as an antidiabetic through studying the effect of plant extract *in vivo* on albino diabetic rats; histopathology was studied to clarify the role of plant extract on pancreatic tissues; haematological studies were used to show the effect of treatment by herb on blood parameters.

## 2. Materials and Methods

### 2.1. Plant Material

The fresh plant sample (Figure 1) was collected in the spring season in the year 2018 from the northern region, Saudi Arabia. The sample was defined in the Biology Department, Faculty of Science, and the authentic sample (FSNBU.C.D.25) was deposited in the Chemistry Department.

### 2.2. Plant Extraction

Plant sample was dried at room temperature, the aerial part was grounded for fine powder, methanol extract was prepared by maceration method, and the plant powder (500 g) was soaked in methanol for 24 hours in a shaker at 25°C. Then, the extract was filtered and stored at −4°C for further investigation [10].

### 2.3. Experimental Animal

150–180 gm weighted adult healthy albino Male rats were used for the experimental study. The animals were housed at regular conditions (temperature, 25 ± 2°C, 55 ± 5% relative humidity, and 12-hour light-dark cycle). Water and a normal diet were allowed to all animals (21% crude protein, 7% crude fiber, 3% fat, 13% moisture, 8% ash, mineral, 1% calcium, 0.5% phosphorus, and 46.3% protein). All experimental procedures were in accordance with the guidelines and instructions of Scientific Research Ethics (COSRE) in *Laboratory of Molecular Genetics* (Egyptian Association for Sustainable Agri.), Egypt (Ethical Approval number: AM/115/01/21).

### 2.4. Experimental Design

Induction of diabetes was done by single intraperitoneal (i.p.) injection of STZ in a dose of 58 mg/kg. Thirty animals were used and divided in to 5 groups (six animals per each):

  Group 1: control group, only saline injection.
  Group 2: diabetic group injected with 58 mg/kg STZ i.p.
  Group 3: diabetic group injected with metformin with 100 mg/kg body weight for 2 weeks.
  Group 4: diabetic group injected with insulin at a dose of 10 U/kg body weight for 2 weeks.
  Group 5: diabetic group injected with plant extract at a dose of 300 mg/kg body weight for 2 weeks.

### 2.5. Toxicity Studies

The OECD guideline no. 420 was used to conduct an acute toxicity test on a plant extract (Organization of Economic Co-operation and Development) according to the methods described by Elsharkawy et al. [11]. At the conclusion of the trial, no fatalities were recorded, and the plant extract was confirmed to be safe up to a dosage of 2,000 mg/kg.

### 2.6. Haematological Study

Blood samples were taken from each rat after the treatment and recovery period. The analysis was done for estimation of hemoglobin concentration according to Drabkin and Austin [12], red blood cells (RBCs) were counted according to Dacie and Lewis [13], and white blood cells (WBCs) were counted according to Mitruka et al. [14].

### 2.7. Histopathological Analysis of the Pancreatic Tissue

The pancreatic tissue samples were fixed in 10% formalin solution for 48 hours before being rinsed under running water for 8 hours for histopathological examination. During the usual tissue control phase, they were treated with alcohol (70°, 80°, 90°, 96°, and 100°) and a succession of xylenes before being blocked in paraffin. On the slides, the samples were produced by cutting 4 *μ*m pieces from each block. They were stained with hematoxylin-eosin (HE) staining and prepared for histopathological examination. A light microscope was used to image and examine the relevant regions (Olympus BX51 optical microscope and Olympus DP25 digital camera, Japan) [15].

### 2.8. UPLC/MS Analysis

The sample (100 *μ*g/mL) solution was prepared using high-performance liquid chromatography (HPLC) analytical grade solvent of MeOH, filtered using a membrane disc filter (0.2 *μ*m), and then subjected to LC-ESI-MS analysis. Sample injection volumes (10 *μ*L) were injected into the UPLC instrument equipped with a reverse phase C-18 column (ACQUITY UPLC-BEH C-18, 1.7 *µ*m particle size—2.1 × 50 mm column). The sample mobile phase was prepared by filtering using a 0.2 *μ*m membrane disc filter and degassed by sonication before injection.

A gradient mobile phase included two eluents: eluent A is H_2_O acidified with 0.1 percent formic acid, and eluent B is MeOH acidified with 0.1 percent formic acid. Mobile phase elution was performed at a flow rate of 0.2 mL/min with a flow rate of 0.2 mL/min. The aforementioned gradient was used for elution. The following parameters were used for the analysis: source temperature of 150°C, cone voltage of 30 eV, capillary voltage of 3 kV, desolvation temperature of 440°C, cone gas flow of 50 L/h, and desolvation gas flow of 900 L/h in negative ion mode. Between m/z 100 and 1000, mass spectra were identified using the ESI negative ion mode. The peaks and the spectra were analyzed using the MassLynx 4.1 software and tentatively recognized by correlating the retention time (Rt) and mass spectrum to the data.

### 2.9. Statistical Analysis

Quantitative data were expressed as the mean ± standard error of means. A paired-sample *t*-test was employed to determine if there were any significant differences between each tested compound with the referenced antifungal drug. The program used was Statistical Package for the Social Sciences (SPSS), version 11.

## 3. Results and Discussion

### 3.1. Toxicity Studies

Oral administration of alcoholic extract of *D. tortuosa* in doses up to 2, 000 mg/kg failed to kill albino Male rats within 24 h. The tested extract is considered highly safe, since substances possessing LD50 higher than 50 mg/kg b.wt. are considered nontoxic [11].

### 3.2. Effect of Herbal Extracts on Blood Glucose Level

Table 1 and Figure 2 show the findings of a two-week investigation on the effects of metformin, insulin, and plant extract on blood glucose levels in normal and diabetic rats subjected to various treatments. Control group showed normal blood glucose level with an average value of 90.6 mg/dl. The diabetic group recorded a significant increase in blood glucose level (541.6 mg/dl), compared with normal controls; similarly, metformin and insulin diabetic-treated groups recorded a substantial fall in the levels of blood glucose (194.8 and 133.8 mg/dl, respectively), compared with the diabetic group. The treatment with plant extract recorded a significant decrease in blood glucose level (284 mg/dl), compared with the diabetic group. Taken into consideration, the treated groups except the insulin group showed significant elevation in blood glucose level.

### 3.3. Effects of Herbal Extracts on Insulin Levels in the Blood

The impacts of metformin, insulin, and herbal extracts on blood insulin levels in normal and diabetic rats subjected to various treatments for 2 weeks are reported in Table 2 and Figure 3. The control group showed a normal blood insulin level with an average value of 1.38 (ng/ml). Meanwhile, diabetic groups recorded a substantial fall (*P* < 0.05) in the level of blood insulin (0.33 ng/ml), when compared with the normal control. Similarly, the metformin-treated group showed no noteworthy growth, while insulin diabetic-treated groups recorded a considerable boost (*P* < 0.05) in blood insulin levels (0.89 and 1.29 ng/ml, respectively) when compared to the normal group. The treatment with herbal extract showed a mild decrease in blood insulin level (0.93 ng/ml) when compared with the normal group.

### 3.4. Effects of Herbal Extracts on Body Weight in Diabetic and Normal Rats

The effects of metformin, insulin, and herbal extracts on body weight in normal and diabetic rats subjected to various treatments for two weeks are summarized in Table 3 and illustrated in Figure 4. Control group showed normal body weight gain with normal increase (12%) during the two weeks of study experiments. Meanwhile diabetic groups recorded a significant decrease (*P* < 0.05) in body weight (17%) when compared with the initial weight. Similarly, the metformin and insulin diabetic-treated groups recorded a significant decrease (*P* < 0.05) in body weight (2.9% and 3.4%, respectively) when compared with the initial weight. The treatment with herbal extracts recorded a significant decrease (*P* < 0.05) in body weight (7.5%) when compared with the initial weight.

### 3.5. Effects of Herbal Extracts on Hemoglobin Concentration, Red Blood Cell Count, and Platelet Count

The control group showed normal RBC count, Hb concentration, and platelet count. The diabetic group recorded a significant decrease (*P* < 0.05) in the RBC count (46.8%), Hb concentration (10.8%), and platelet count (37.4%) when compared with the corresponding control values.

Similarly, the metformin and insulin diabetic-treated groups recorded a noteworthy upsurge (*P* < 0.05) in the RBC count (98.4% and 84.03%, respectively), the Hb concentration in metformin and insulin diabetic-treated groups recorded no significant change (1.4% and −2.8%, respectively), and platelet count in metformin diabetic-treated group recorded no significant increase (36.7%), while the insulin diabetic-treated groups recorded significant increase (54.7%) when compared with the corresponding values in the diabetic group. The treatment with herbal extract exhibited a substantial increase (*P* < 0.05) in the count of RBCs (80.7%); finally, the platelet count showed a significant decrease in the herb by about 76.4%, when compared with the corresponding values in the diabetic-treated group as shown in Table 4 and Figures 5–7.

### 3.6. Effects of Herbal Extracts on the White Blood Cell (WBC) Count in Normal and Diabetic Rats Exposed to Different Treatments

The effect of methanol extract of *D. tortuosa* on WBC count is illustrated in Table 5 and Figure 8. The diabetic group recorded a considerable decline (*P* < 0.05) in WBC quantities (46.01%) when compared with the corresponding control values. Similarly, the metformin and insulin diabetic-treated groups recorded a substantial increase (*P* < 0.05) in the count of WBCs (118.03% and 95.1%, respectively) when compared with the corresponding diabetic groups. The treatment with plant extract recorded a substantial increase (*P* < 0.05) in WBCs (78.7%) when compared with the corresponding diabetic groups.

### 3.7. Histopathological Study of the Pancreas

Figure 9 shows the histopathological structure of pancreatic tissue. The pancreatic B cell of Group 2 diabetic rats was completely damaged compared to control Group 1 due to STZ induction, and it was discovered that, after treatment with methanol extract of *D. tortuosa*, the atrophy of Langerhans islets, degeneration, and apoptosis by B cell decreased, and pancreatic structure was restored in diabetic rats. Additionally, metformin treatment changed the pancreatic structure.

### 3.8. UPLC-QTOF/ESI-MS Screening

Ultraperformance liquid chromatography in combination with mass spectrometry method was deployed to examine the phytochemical components in plant extract, the phenolic fraction of methanol extract was analyzed by UPLC/ESI-MS, phytochemical screening of plant extract revealed the presence of a high amount of flavonoid compounds, and this was confirmed by identification of flavonoid, flavonoid glucoside, and phenolic acid by using positive mode (+) ESI-Ms, and the identification of compounds was determined on the basis of the pattern of mass fragments and ion response. Compounds were identified as listed in Table 6, and chromatograms are presented in Figure 10. Molecular formula and molecular weight were compared with [16, 17].

The chemical was identified using literature data to compare the molecular ion peak (M-H) and fragmentation patterns derived from MS/MS [18, 19]. From the fragmentation pattern, the simple regular cleavage of glucoside bonds in the molecular ion peaks [M-H] can be concluded, as an example in the spectra of flavonol-3-glucoside; the successive loss of a glycone gives fragment ion at 315, (314) m/z 285 (284), m/z, 151 (isorhamnetin), fragment ion peak at 315 due to loss of glucoside, and fragment ion at 301 [315-CH3) due to loss of methyl group, while fragmentation of 301 through MS/MS gives three fragment peaks (257 [M-CO2], 171, and 151) [20]. Kaempferol gives fragmentation pattern (284 [M-H], 255, 179, 151) despite homiletic cleavage of B ring [18].

## 4. Discussion

*D. tortuosa* is used as a traditional medicinal plant in Egypt and Saudi Arabia. The current study was assumed to examine the antidiabetic activity of methanol extract of the plant. Diabetes is a common disease spread in Arabian countries and the world affecting the major population. It is a metabolic disease, causing complication in many organs such as liver, kidney, and pancreas [21]. An experimental model was designed to examine how antidiabetic agents affect diabetes; STZ is used for experimental diabetes which has toxic effects on pancreatic beta cells and causes oxidant effects and the formation of nitric acid together with DNA damage. The results of this experimental study show that the plant extract exhibits significant antihyperglycemic activity at a dose level of 300 mg\kg. An increase of glucose level in blood induces the excretion of insulin which controls the production of glucose [22].

The diagnosis of diabetes on male Wister albino rats was confirmed by increased serum glucose level after 28 days of injection of STZ in diabetic rats. The serum glucose level was measured as 541.5 ± 15.39 mg/dL in Group 2, as compared with the nondiabetic rats (control group). It was observed that the glucose levels of Groups 3 and 4 decrease, while the glucose levels of Group 5 were higher than those of Groups 3 and 4 but lower than those of Group 2 (STZ). The serum insulin level of Group 1 was 34.88 ± 0.36 mg/dl. The serum insulin level of the STZ induced rats (Group 2) was lower than that of Group 1 (0.33 ± 0.06 mg/dl), while the herb (Group 5) showed a decrease in serum insulin level (0.93 ± 0.11 mg/dl) more than Group 3 (metformin). This is common and agrees with a pervious study on Apiaceae family used to treat diabetes [23].

Flavonoid compounds have many biological activities; for example, they protect the body against oxidative stress. Flavonoid-rich food reduces the risk of oxidative compounds [24, 25]. Isorhamnetin glycoside and kaempferol possess an antidiabetic effect and influence lipid content. Rutin showed a significantly lower level of plasma glucose and increased insulin level at 10 mg/kg in a previous study on diabetic mice [26]. There are many previous studies on antidiabetic activity of flavonoid compounds, which revealed the role of flavonoid compounds in the treatment of diabetes by different mechanisms. Most significant mechanisms are decreasing insulin resistance, inflammation, and oxidative stress in muscle by increasing insulin production, reducing apoptosis, and boosting profanation of pancreatic B cells [27]. The previous studies agreed with this study where the major compounds of a phenolic fraction rutin, kaempferol, and isorhamnetin-3-O-rutinoside which have the potential antidiabetic effect, reflecting the role of the plant as an antidiabetic drug.

Study of the effect of a phenolic fraction on haematological parameters showed a decrease in RBCs, Hb content, and platelet count in diabetic rats, and this decrease in RBCs and Hb indicated the rats suffer from anemia, as a result of the toxic effect of STZ. Meanwhile the treatment with herbal extract exhibited a significant increase in the RBC count (80.7%). The platelet count showed a significant decrease in the herb-treated group, by approximately 76.4% when compared with the corresponding values in the diabetic-treated group, while there was no significant change in Hb concentration compared with the diabetic group. Current studies came to agree with other previous studies by Helal et al. [28] and were contradictory with Hadiya [29] who found that *Nigella sativa* extract caused significant increase in hemoglobin and platelet counts. The plant *D. tortuosa* in this study can be used as an antidiabetic drug and we recommended following the study on this plant.

## 5. Conclusion

In the current study, a glucose induction hyperglycemic model was selected to monitor the antihyperglycemic activity of plant extract. The results concluded that methanol extract of *D. tortuosa* decreases the blood glucose level and improves blood parameters, increasing WBCs and RBCs compared with the diabetic group. The extract also inhibits histopathological changes induced in the pancreas of diabetes group. Phytochemical screening by HPLC/MS of flavonoid fraction revealed the presence of more than 20 peaks; 12 peaks were identified by comparison with literature data. The major flavonoid compounds rutin, kaempferol and isorhamnetin-3-O-rutinoside confirmed the role of the plant as an antidiabetic because these compounds have antioxidant activity and decrease the oxidative stress, which is considered as one of the most important reasons for the pancreatic damage. These obtained results support the use of the plant in antidiabetic traditional preparations after further studies.

## Figures and Tables

**Figure 1:** Picture of plant *Deverra tortuosa*.

**Figure 2:** Effects of metformin, insulin, and herbal extract on the blood glucose level in normal and diabetic rats. ^a^Significantly different from control at *P* ≤ 0.05. ^b^Significantly different from STZ at *P* ≤ 0.05.

**Figure 3:** Effects of metformin, insulin, and herbal extract on the blood insulin level in normal and diabetic rats. ^a^Significantly different from control at *P* ≤ 0.05. ^b^Significantly different from STZ at *P* ≤ 0.05.

**Figure 4:** Effects of metformin, insulin, and herbal extract on percentage change in the body weight in normal and diabetic rats. ^a^Significantly different from control at *P* ≤ 0.05. ^b^Significantly different from STZ at *P* ≤ 0.05.

**Figure 5:** Effects of metformin, insulin, and herbal extract on the RBC count in normal and diabetic rats. ^a^Significantly different from control at *P* ≤ 0.05. ^b^Significantly different from STZ at *P* ≤ 0.05.

**Figure 6:** Effects of metformin, insulin, and herbal extract on the Hb concentration in normal and diabetic rats. Data are presented as means ± SEM, *n* = 6. ^a^Significantly different from control at *P* ≤ 0.05. ^b^Significantly different from STZ at *P* ≤ 0.05.

**Figure 7:** Effects of metformin, insulin, and herbal extract on the platelet count in normal and diabetic rats. Data are presented as means ± SEM, *n* = 6. ^a^Significantly different from control at *P* ≤ 0.05. ^b^Significantly different from STZ at *P* ≤ 0.05.

**Figure 8:** Effects of metformin, insulin, and herbal extract on the WBC count in normal and diabetic rats. ^a^Significantly different from control at *P* ≤ 0.05. ^b^Significantly different from STZ at *P* ≤ 0.05.

**Figure 9:** Histopathological structure of the normal pancreas. (a) The normal pancreas showing average-sized normocellular islets with predominating beta cells (black arrow) and less frequently alpha cells in the periphery (blue arrow), average intervening blood capillaries (yellow arrow), and average exocrine areas (red arrow) (H&E ×400). (b) The diabetic pancreas showing relatively small-sized islets with apoptotic beta cells (black arrow), excess alpha cells (red arrow), average intervening blood capillaries (blue arrow), and average exocrine areas (yellow arrow) (H&E ×400). (c) The metformin-treated pancreas showing average islet with average beta cells (red arrow), mildly dilated intervening blood capillaries (blue arrow), average exocrine areas (yellow arrow), and mildly congested blood vessels (black arrow) (H&E ×400). (d) The insulin-treated group showing relatively small-sized pale-staining islets of Langerhans (black arrow) and average exocrine areas (yellow arrow) (H&E ×200). (e) Herb treatment showing hypocellular islets with scattered beta cells (black arrow) with mildly dilated intervening blood capillaries (blue arrow) and average exocrine areas (yellow arrow) (H&E ×400).

**Figure 10:** LC-MS chromatogram of the methanol extract of *D. tortuosa*.

**Table 1:** Effect of metformin, insulin, and plant extract on blood glucose level.

Groups	Blood glucose level (mg/dl)
Control G1	90.6 ± 5.9
STZ G2	541.5 ± 15.39^a^
STZ + met (G3)	194.8 ± 12.8^a, b^
STZ + insulin (G4)	133.8 ± 12.46^b^
STZ + herb (G5)	284 ± 19.9^a, b^

Data are presented as means ± SEM (*n* = 6). ^a^Significantly different from control at *P* ≤ 0.05. ^b^Significantly different from STZ at *P* ≤ 0.01.

**Table 2:** Effects of metformin, insulin, and herbal extract on the blood insulin level in normal and diabetic rats.

Groups	Blood insulin level (mg/dl)
Control	1.38 ± 0.17
STZ	0.33 ± 0.06^a^
STZ + met	0.89 ± 0.14
STZ + insulin	1.29 ± 0.17^b^
STZ + herb	0.93 ± 0.11

Data are presented as means ± SEM (*n* = 6). ^a^Significantly different from control at *P* ≤ 0.05. ^b^Significantly different from STZ at *P* ≤ 0.01.

**Table 3:** Effects of metformin, insulin, and herbal extract on the percentage change in body weight in normal and diabetic rats.

Groups	Percentage change in body weight
Control	11.83 ± 1.6
STZ	−16.83 ± 2.15
STZ + met	−3.00 ± 4.29
STZ + insulin	−3.66 ± 1.20
STZ + herb	−7.00 ± 2.59

Data are presented as means ± SEM (*n* = 6). ^a^Significantly different from control at *P* ≤ 0.05. ^b^Significantly different from STZ at *P* ≤ 0.01.

**Table 4:** Effects of metformin, insulin, and plant extract on RBC count, Hb concentration, and platelet count in normal and diabetic-treated rats.

Groups	Parameters					
	RBC count (10^6^/*µ*l)		Hb concentration (g/dl)		Platelet count (10^3^/*µ*l)	
	Mean ± SE	%	Mean ± SE	%	Mean ± SE	%
Control	7.18 ± 0.16	—	15.83 ± 0.23	—	578 ± 20	—
STZ	3.82 ± 0.003^a^	−46.8	14.10 ± 0.03^a^	−10	362 ± 0.36^a^	−37
STZ + met	7.58 ± 0.003^b^	98.4	14.33 ± 0.07^a^	1.4	495 ± 16	36.7
STZ + insulin	7.03 ± 0.14^b^	84.03	13.77 ± 0.24^a^	−2.8	560 ± 17^b^	54.7
STZ + herb B	6.90 ± 0.44^b^	80.7	14.00 ± 0.48^a^	−0.7	339 ± 2.8^a^	−6.4

RBC, red blood cell; Hb, hemoglobin. ^a^Significantly different from control at *P* ≤ 0.05. ^b^Significantly different from STZ at *P* ≤ 0.01.

**Table 5:** Effects of metformin, insulin, and herbal extract on WBC count in normal and diabetic rats exposed to different treatments.

Groups	WBCs (10^3^/*µ*l)
Control	11.33 ± 0.14
STZ	6.10 ± 0.036^a^
STZ + met	13.33 ± 2.13^b^
STZ + insulin	11.90 ± 1.18^b^
STZ + herb	10.90 ± 0.56^b^

Data are presented as means ± SEM (*n* = 6). ^a^Significantly different from control at *P* ≤ 0.05. ^b^Significantly different from STZ at *P* ≤ 0.01.

**Table 6:** Compounds identified from the phenolic fraction of *D. tortuosa* by the HPLC-MS negative mode.

No.	Rt (min)				Identified compound (M)
		%	[M-H]^−^	MS/MS	
1	5.62	3.2	299	MS2 [137]: (100) [M-H-Glc], 93 [M-H-Glc-CO2]	4-Hydroxybenzoic acid 4-O-glucoside
2	7.44	6.18	477	MS2 [301]: (100), 151, 135	Quercetin 3-O-glucuronide
3	9.28	2.20	341	303, 257, 193	Hesperidin derivative (342)
4	9.63	1.04	447	MS2 [447]: 429 (2), 415 (2), 285 (100); MS3 [285]: 270 (100), 257 (4), 253 (40), 229 (5), 225 (16), 137 (5)	Kaempferol glucoside
5	15.65	5.6	447	MS2 [300.9]: 178.8, 150.8, 106.9, 120.8, 272.9, 228.9, 256.8	Quercetin 3-O-*β*-rhamnoside
6	20.25	7.5	593	MS2: 285 (100), 257 (22) MS3 [593 ⟶ 285]: 257	Kaempferol-3-O-rutinoside
7	23.76	8.08	301	257 (9100), 247, 201	Quercetin
8	24.6	8.25	609	300 (100), 271, 255, 151	Rutin
9	26.57	102.5	623	315 (100), 300, 271, 255	Isorhamnetin-3-O-rutinoside
10	27.60	5.62	316	MS2 [301] (100), 272, 256, 154, 107	Isorhamnetin
11	28.03	1.78	179	MS2: 161 (100), 135	Caffeic acid
12	31.27	15.5	285	239, 69 (100), 187.22, 143.21	Kaempferol

## Data Availability

Data are available upon request to the corresponding author.
